# The Value of Serum Exosomal miR-184 in the Diagnosis of NSCLC

This article has been retracted.

**DOI:** 10.1155/2022/9713218

**Published:** 2022-04-11

**Authors:** Shujun Li, Yanming Lin, Yanxia Wu, Hualin Chen, Zhong Huang, Muwen Lin, Jiali Dong, Yongcun Wang, Zhixiong Yang

**Affiliations:** ^1^Department of Pulmonary Oncology, Affiliated Hospital of Guangdong Medical University, Zhanjiang 524023, China; ^2^Guangdong Medical University Affiliated Pathology Diagnosis and Research Center, Zhanjuang 524023, China

## Abstract

Lung cancer has the highest morbidity rate (11.6%) and mortality rate (18.4%) among all current tumors. The morbidity rate in China accounts for approximately one-third, and it is still rising. Nonsmall cell lung cancer is the most common type of lung cancer, accounting for 80%–85% of all lung cancers, and approximately 57% of patients with advanced nonsmall cell lung cancer have distant metastases at the time of diagnosis. To explore the expression changes in microRNA-184 (miR-184) and its clinical value in serum exosomes of patients with nonsmall cell lung cancer (NSCLC). This study adopted a case-control study method, selecting 88 patients (NSCLC group) from June 2015 to June 2017 in our hospital who are confirmed to have NSCLC by fiber-optic bronchoscopy, and 90 patients who are confirmed to have benign lung diseases by pathological examination during the same period (control group). Fluorescence quantitative PCR technology is used to detect the levels of miR-184 in serum exosomes of the two groups, and the differences in the levels of miR-184 in serum exosomes of NSCLC patients with different pathological characteristics are analyzed. According to the results of the 3-year follow-up, the miR-184 levels in serum exosomes of NSCLC patients are grouped and compared. The expression level of miR-184 in serum exosomes in the NSCLC group is significantly higher than that in the control group, and the difference between the two groups is statistically significant (*p* < 0.05). The ROC curve is drawn with the expression level of miR-184 in serum exosomes of the two groups of patients. The results showed that the area under the ROC curve for the differential diagnosis of NSCLC and benign lung tumors with the expression level of miR-184 in serum exosomes is 0.927, and the sensitivity is 87.61%, while the specificity is 84.02%. The expression levels of miR-184 in serum exosomes of NSCLC patients with different pathological characteristics, in different TNM stages [(I+II) vs. (III+IV)], lymph node metastasis (yes vs. no), and different degrees of differentiation [(High + Medium) vs. Poorly differentiated] are compared and showed statistical significance (*p* < 0.05). In 88 NSCLC patients, after 3 years of follow-up, 33 survived, and 55 died, with a survival rate of 37.50%. The expression of miR-184 in serum exosomes of the 33 surviving patients is significantly lower than that of the nonsurviving group (*p* < 0.05). The expression level of miR-184 in serum exosomes of NSCLC patients is significantly increased, which has a certain value for the differential diagnosis of the nature of benign and malignant lung diseases and is closely related to the prognosis of patients.

## 1. Introduction

This study included NSCLC cases and explored the relationship between the level of miR-184 and the development of NSCLC and is expected to provide clinical evidence for patient prognosis. Nonsmall cell lung cancer (NSCLC) is the most common type of lung cancer, accounting for approximately 80% of all types of lung cancer [1]. The survival rate of patients is low, and the prognosis is also poor. To diagnose NSCLC as soon as possible and improve the survival rate of patients, it is very important to study the mechanism of NSCLC. There have been many studies on the mechanism of NSCLC, but controversies remain. Our goal is to provide new ideas for clinical treatment and ultimately to identify specific targeted drugs [2, 3].

MicroRNAs (microRNAs, miRNAs) are widely involved in the biological processes of cells, and the expression of some miRNAs is tissue-specific. Therefore, changes in the expression of miRNAs can be used to assess the occurrence and development of diseases [4]. According to previous studies, some miRNAs play important roles in the occurrence and development of NSCLC. The miRNAs miR-100, miR-145, and miR-223 have different properties in different tumors and can be oncogenes or tumor suppressor genes [5, 6]. Previous studies have found that miR-184 is overexpressed in kidney cancer tissues and is closely related to the degrees of tumor differentiation and tumor metastasis and to patient prognosis. Analysis of miR-184 may reveal the effects on the expression of related proteins that cause the abnormal proliferation and metastasis of tumor cells [7, 8]. Combined with a large amount of clinical research data, it is speculated that miR-184 may also be related to the occurrence and development of NSCLC, and the outcome of patients can be predicted by the level of miR-184. Recent studies have found that some miRNAs can cause drug resistance in targeted therapy and influence the therapeutic effect.

As described in the literature [9, 10], exosomes can mediate the transfer of miRNAs and stabilize them in the circulatory system. Because the expression of miRNAs in lung cancer is not the same, serum exosome miRNAs have the conditions to become tumor biomarkers. We used real-time fluorescence quantitative PCR to detect the expression level of serum exosomal miRNA-184 in patients with NSCLC and patients with benign lung diseases and explored the diagnostic efficacy of serum exosomal miRNA-184 in NSCLC and its effect on benign and malignant lesions.

## 2. Medicines and Detection Method

This study adopted a case-control study method, selecting 88 patients (NSCLC group) who are confirmed to have NSCLC by fiber-optic bronchoscopy from June 2015 to June 2017 in our hospital and 90 patients who are confirmed to have benign lung diseases by pathological examination during the same period (control group).

Inclusion criteria: (1) the age range of patients is 47–82 years; (2) the diagnostic criteria of NSCLC patients referred to the standards in the “2011 NCCN Guidelines for the Diagnosis and Treatment of Nonsmall Cell Lung Cancer” [11]; (3) in the diagnosis of patients with NSCLC or benign lung diseases, the diagnostic results are confirmed by pathological examination; and (4) NSCLC patients are followed up for at least 3 years, and the outcome data are complete. Exclusion criteria: (1) metastatic lung cancer; (2) patients with recurrence after lung cancer surgery; (3) lung cancer patients who had received chemotherapy, radiotherapy or immunotherapy; (4) malignant tumors at other sites; and (5) accompanied by HIV infection, Rheumatic immunological diseases.

The 7500 real-time quantitative reverse transcription-polymerase chain reaction instrument, reverse transcription kit, and qPCR kit are purchased from Applied Biological Systems (ABI, USA), the exosome extraction kit is purchased from SBI, the JEM-100cxII transmission electron microscope is purchased from Japan Electronics Corporation, the spectrophotometer is purchased from Bo Le Biomedical Products (Shanghai) Co., Ltd., and the total RNA extraction reagent (TRIzol) reagent is purchased from Invitrogen.

Blood samples are collected from all subjects, and centrifugation is performed to obtain the serum. Serum exosomes are extracted and identified following the operating instructions of the SBI Exosome Extraction Kit. After staining the processed sample, it is observed under an electron microscope to observe the particle shape, and a NanoSight NS300 instrument is used to determine its concentration. The sample is diluted as required to make the concentration in the range of 108∼109/ml, and the instrument threshold is set to 5.

TRIzol reagent is used to lyse the exosomal sample, and the total RNA of the sample is extracted. The sample is first purified with a silica gel mold adsorption column so that the sample met the detection standard. After reaching the detection standard, the cDNA sample is obtained and subjected to reverse transcription (reaction conditions: 16°C for 15 min, 42°C for 60 min, 85°C for 5 min, 4°C for 5 min). The fluorescent dye incorporation method is used to quantitatively detect the level of miRNA-184 in exosomes. The formulas are miRNA-184 expression level = 2^-△△Ct^, with miRNA-39 as the external reference gene, ∆Ct = CtmiRNA-184-CtmiRNA-39 [12].

In this paper, the expression level of miR-184 and other measurement indicators are tested by the normal distribution, and they all conformed to the approximate normal distribution or the normal distribution, which is expressed by ($\bar{X}$ ± *s*) [13–16]. The *t*-test is used for comparisons between the two groups. Enumeration data are expressed as percentages, and the comparison is performed by the *χ*^2^ test. The survival analysis is performed by the Kaplan-Meier method. The diagnostic analysis adopted the receiver operating curve (ROC) method for analysis. SPSS 21.0 software is used for data processing, and the inspection level is *α* = 0.05.

## 3. The Experimental Result

### 3.1. Comparison of the General Information of the Two Groups of Patients

Comparing age, sex, smoking, alcohol consumption, diabetes, hypertension, and abnormal blood lipid levels between the NSCLC group and the control group, there are no statistically significant differences between the two groups (*P* > 0.05) [17–20].  Table 1 is comparison of general data between the two patient groups.

### 3.2. Comparison of the miR-184 Expression Levels in Serum Exosomes of the Two Groups of Patients

The expression level of miR-184 in serum exosomes of the NSCLC group is significantly higher than that of the control group, and the difference between the two groups is statistically significant (*p* < 0.05).  Table 2 is comparison of miR-184 expression levels in serum exosomes of two groups of patients.  Figure 1 shows histogram of miR-184 expression levels in serum exosomes of two groups of patients.

### 3.3. Value of miR-184 Expression in Serum Exosomes in the Differential Diagnosis of NSCLC and Benign Lung Diseases

The ROC curve is drawn for the miR-184 expression levels in serum exosomes of the two groups of patients. The results showed that the area under the ROC curve for the differential diagnosis of NSCLC and benign lung tumors with the expression level of miR-184 in serum exosomes is 0.927, the sensitivity is 87.61% and the specificity is 84.02%.  Figure 2 presents ROC curve of miR-184 expression level in serum exosomes for differential diagnosis of NSCLC and benign lung diseases.

### 3.4. Relationship between the Expression of miR-184 in Serum Exosomes and the Pathological Characteristics of NSCLC Patients

Comparing the miR-184 expression levels in serum exosomes of NSCLC patients with different pathological characteristics, in different TNM stages [(I+II) vs. (III+IV)], lymph node metastasis (yes vs. no), and degree of differentiation [(High + Medium) vs. Poorly differentiated], the difference is statistically significant (*p* < 0.05).  Table 3 is the relationship between the expression of miR-184 in serum exosomes and the pathological characteristics of NSCLC patients.

### 3.5. Relationship between the Expression of miR-184 in Serum Exosomes and the Prognosis of NSCLC Patients

After 3 years of follow-up for 88 patients with NSCLC, 33 survived, and 55 died, for a survival rate of 37.50%. The survival curve is shown in Figure 3. Among the 33 surviving patients, the expression of miR-184 in serum exosomes is significantly lower than that in the group of patients who died, and the difference is statistically significant (*p* < 0.05). Figure 3 shows 3-year survival curve of 88 patients with NSCLC.  Table 4 is differences in the expression of miR-184 in serum exosomes of patients with different prognostic outcomes.

## 4. Data Analysis and Result Discussion

Although some miRNAs have been proven to have diagnostic value for NSCLC, they are generally based on the expression of miRNAs in tumor tissues or cells. The detection of miRNA in tumor tissue requires invasive surgery or puncture operations, which is not conducive to widespread use. Human serum can be used as an miRNA test sample, but the serum composition is more complicated. If the source is confused, the test results may be affected. Data show that serum exosomes are simpler and easier to obtain than serum exosomes, as it involves a noninvasive operation, and the sample also contains some miRNAs for testing, which are currently receiving extensive clinical attention and are expected to become a new research direction. At present, only a few studies have proposed that exosomal miRNA-184 is involved in the occurrence and development of NSCLC, and the expression profiles of miRNA molecules in exosomes and the total miRNA molecules in blood are significantly different. Thus, the research remains controversial. Based on previous studies, this study included patients with benign and malignant diseases to explore the clinical efficacy of miR-184 expression in serum exosomes in the differential diagnosis of benign and malignant lung diseases.

The results of this study showed that the expression level of serum exosome miR-184 in the NSCLC group is significantly higher than that in the control group. The level of miR-184 in serum exosomes had good sensitivity and specificity for distinguishing benign and malignant lung diseases. These results indicate that serum exosome miR-184 is expected to become a diagnostic marker for NSCLC. The reason for the analysis is that exosomal miR-184 acts as a messenger of intercellular information, mediates the tumor microenvironment by participating in the transmission of information and participates in the occurrence and development of tumors to a certain extent. When a tumor appears, the number of exosomes secreted by tumor cells is greater than that secreted by normal cells. There is a significant difference in the expression profiles of miR-184 in exosomes derived from tumor cells and exosomes secreted by normal cells. Therefore, the expression level of miR-184 in exosomes can be used as a diagnostic marker for NSCLC and can differentiate it from other benign diseases.

The results of this study showed that the expression levels of miR-184 in serum exosomes of NSCLC patients with different pathological characteristics are significantly different. The reason for the analysis is that the surface proteins of exosomes can bind to the receptor cells, mediate interactions between the receptor and the ligand and transfer the contents of the exosomes to the target through endocytosis, exocytosis or cell membrane fusion. In the cell, these contents affect the structure and environment of the target cell and ultimately affect its function. When tumors occur, exosomes transport miR-184 and oncogene-related bioactive molecules to tissue cells, which affects the biological process of tumors. The expression level of miR-184 is positively correlated with the degree of tumor development. Based on the results of this study, it is speculated that miR-184 can activate the Wnt/*β*-catenin signaling pathway in cells. In addition, miR-184 may also affect the process of epithelial cell mesenchymal transformation, eventually inducing the formation of tumor stem cells and promoting tumor invasion and metastasis.

The results of this study showed that the expression level of serum exosome miR-184 in the survival group is significantly lower than that in the death group. The serum exosomal miR-184 level can be used as a predictor of patient prognosis. Studies have shown that miRNAs can regulate the rapid deadenylation of the mRNA of their target genes, leading to rapid attenuation of mRNA and lower expression levels, thereby playing a regulatory role. The abnormally high expression of miR-184 promotes the occurrence and development of NSCLC, and miR-184 may also be involved in the regulation of multiple signaling pathways in the biological process of lung cancer. The promoter region of miR-184 is hypomethylated, which induces a large amount of miR-184 expression. Highly expressed miR-184 may promote the metastasis of cancer cells through tumorigenesis-related mechanisms and ultimately lead to the poor prognosis of NSCLC patients.

## 5. Conclusion

In summary, the expression level of miR-184 in serum exosomes of NSCLC patients is significantly increased, which has a certain value for the differential diagnosis of the nature of benign and malignant lung diseases and is closely related to the prognosis of patients.

miRNAs are involved in a variety of life processes, such as embryonic development, cell proliferation, apoptosis, metabolism and even tumor biological processes. Future research can focus on promoting or inhibiting the expression of miRNAs related to exosomes, analyzing the expression characteristics of miRNAs related to the occurrence and development of NSCLC through ROC curve analysis, improving the sensitivity and specificity of diagnosing NSCLC, and guiding the clinic in implementing timely treatment measures, thus reducing the mortality of lung cancer and improving the prognosis of patients.

## Figures and Tables

**Figure 1:** Histogram of miR-184 expression levels in serum exosomes of two groups of patients.

**Figure 2:** ROC curve of miR-184 expression level in serum exosomes for differential diagnosis of NSCLC and benign lung diseases.

**Figure 3:** 3-year survival curve of 88 patients with NSCLC.

**Table 1:** Comparison of general data between the two patient groups.

Normal information	NSCLC group (*n* = 88)	Control group (*n* = 90)	t/*χ*^2^	*P*
Age			1.079	0.299
≥60	47 (53.41)	55 (61.11)		
<60	41 (46.59)	35 (38.89)		
Gender (%)			0.618	0.432
Male	54 (61.36)	50 (55.56)		
Female	34 (38.64)	40 (44.44)		
Smoking (%)			0.349	0.555
Yes	43 (48.86)	40 (44.44)		
No	45 (51.14)	50 (55.56)		
Drinking (%)			1.173	0.279
Yes	34 (38.64)	42 (46.67)		
No	54 (61.36)	48 (53.33)		
Diabetes (%)			1.381	0.240
Yes	14 (15.91)	9 (10)		
No	74 (84.09)	81 (90)		
High blood pressure(%)			1.169	0.280
Yes	17 (19.32)	12 (13.33)		
No	71 (80.68)	78 (86.67)		
Dyslipidemia (%)			1.302	0.254
Yes	18 (20.45)	25 (27.78)		
No	70 (79.55)	65 (72.22)		

**Table 2:** Comparison of miR-184 expression levels in serum exosomes of two groups of patients ($\bar{X}$ ± *s*, 2^-△△ct^).

Group	n	miR-184	t	*p*
NSCLC group	88	1.209 ± 0.304	15.054	≤0.001
Control group	90	0.667 ± 0.154		

**Table 3:** The relationship between the expression of miR-184 in serum exosomes and the pathological characteristics of NSCLC patients ($\bar{X}$ ± *s*, 2^-△△ct^).

TNM staging	n	miR-184	t	*p*
I+II	54	1.008 ± 0.278	−8.275	≤0.001
III+IV	34	1.528 ± 0.301		
Lymph node metastasis			4.340	≤0.001
Yes	36	1.371 ± 0.284		
No	52	1.097 ± 0.296		
Pathology type			−1.066	0.290
Adenocarcinoma	70	1.193 ± 0.281		
Others	18	1.271 ± 0.260		
Lesion diameter			0.984	0.328
≥2.0 cm	39	1.241 ± 0.254		
<2.0 cm	49	1.184 ± 0.282		
Differentiation			−8.375	≤0.001
High + middle	51	1.007 ± 0.247		
Poorly differentiated	37	1.487 ± 0.289		

**Table 4:** Differences in the expression of miR-184 in serum exosomes of patients with different prognostic outcomes ($\bar{X}$ ± *s*, 2^-△△ct^).

Prognosis	n	miR-184	t	*p*
Survive	33	0.996 ± 0.289	−5.525	≤0.001
Decease	55	1.337 ± 0.275		

## Data Availability

The data used to support the findings of this study are available from the author upon request.
